# Analysis of N6-Methyladenosine RNA Methylation Regulators in Diagnosis and Distinct Molecular Subtypes of Ankylosing Spondylitis

**DOI:** 10.1155/2022/4942599

**Published:** 2022-09-16

**Authors:** Cheng Zhong, Jia-hua Liang, Zhen Chen, Li-ping Zhong, Guo-dong Sun, Wei-xing Xie, Dong-ping Wang, Wen-de Zhuang, Hao-hua Guo, Da-xiang Jin, Yu-ming Li

**Affiliations:** ^1^Department of Orthopedics, The First Clinical Medical College of Guangzhou University of Chinese Medicine, Guangzhou, China; ^2^Department of Orthopedics, Jiangmen Hospital of Traditional Chinese Medicine Affiliated to Jinan University, Jiangmen, China; ^3^Department of Pancreato-Biliary Surgery, The First Affiliated Hospital, Sun Yat-sen University, Guangzhou, China; ^4^Department of Orthopedics, The First Dongguan Affiliated Hospital of Guangdong Medical University, Dongguan, China; ^5^Department of Orthopedics, The First Affiliated Hospital of Jinan University, Guangzhou, China; ^6^Department of Orthopedics, The First Affiliated Hospital of Guangzhou University of Chinese Medicine, Guangzhou, China

## Abstract

The most frequent internal modification in eukaryotic mRNA is N6-methyladenosine (m6A). However, what we know about the m6A regulators in Ankylosing spondylitis (AS) is still limited. In our study, eight distinct m6A regulators were selected utilizing Differentially Expressed Gene (DEG) analysis of the Gene Expression Omnibus GSE73754 dataset for making comparisons between AS (Ankylosing spondylitis) and non-AS patients. The random forest model and the nomogram model were used to screen the eight candidate m6A regulators and evaluate their prediction accuracy for the occurrence of AS. Furthermore, based on the selected m6A regulators, the AS patients were divided into two subgroups, and we applied principal component analysis algorithms to calculate their m6A score and evaluate the m6A patterns. Our findings revealed that patients in cluster A were linked to activated CD4 T cell immunity and activated CD8 T cell immunity. With its major contributions in the area of immunology, our research in m6A patterns may benefit the future diagnosis and treatment strategies of AS.

## 1. Introduction

Ankylosing spondylitis (AS), also known as radiographic axial spondyloarthritis (already developed structural damage in the sacroiliac joints or spine visible on radiographs), is a chronic inflammatory disease categorized within spondyloarthropathies (SpA) and manifested by damage to the axial skeleton [1]. In the general population, the prevalence of AS ranges from 9 to 30 per 10,000 in the world [2]. Up to 90% of patients with AS have the Human Leukocyte Antigen (HLA)-B27 gene haplotype, while this number in the general population is less than 10%, which indicates that AS has a strong association with the HLA-B27 gene [3]. AS tends to occur in young adults aged 15 to 30. About 80% of its cases first develop before 30 [4]. Up to 15% of patients with AS first have symptoms before 16 years old [5]. The clinical manifestations of AS include arthritis in peripheral joints or peripheral entheses at some point in the disease course. Peripheral arthritis, enthesitis, or dactylitis are involved in the significant clinical manifestation of AS [6]. A single anteroposterior pelvis X-ray, magnetic resonance imaging, ultrasonography, laboratory tests (such as erythrocyte sedimentation rate and C-reactive protein), and HLA-B27 in the patient with clinical features of SpA are beneficial to the diagnosis of AS [7]. The most crucial factor is the presence of HLA-B27 [3]. However, HLA-B60, HLA-B61, HLA-DR8, HLADRB1, and MICA (MHC class I chain-related gene A) play an essential role in AS [8–12]. Moreover, non-HLA susceptibility genes (*PUM1* and *ZFP91)* play a critical role in the development of AS [13]. In addition to IL23R, several risk genes (*TYK2, CARD9, IL12B, IL27, NKX2,* and *PTGER4*) identified in AS are either directly involved in the IL-23–IL-17 pathway or interactive with it [14–18]. The average delay from symptom onset to AS physician diagnosis is 5-7 years [19]. As a result, early screening and effective prevention of AS, from the perspective of genetics, will have a big impact on controlling the number of AS patients.

More than 100 types of RNA modification have been described thus far [20], including 1-methyladenosine, 2-methylthio-N6-isopentenyladenosine, and N6-methyladenosine (m6A) [21]. The most common and abundant internal modification in eukaryotic mRNA is N6-methyladenosine (m6A), which methylates the nitrogen-6 position of adenosine in mRNA via various m6A modification regulators [22]. The primary role of m6A in AS is achieved through the regulation of various immune cells and bone cells [13]. The m6A modification involves three types of regulators, known as “Writers”, “Erasers”, and “Readers” [23]. “Writers”, also named m6A methyltransferases, can be removed by the demethylases or “Erasers”. The m6A modification is recognized by m6A-binding proteins, known as “Readers” [24].

However, the roles of m6A regulators in AS remain limited in scientific and clinical studies. In this study, a microarray dataset from GEO database was used to evaluate the functions of m6A regulators in the diagnosis and subtype classification of AS. Furthermore, the current study provides more insight into how m6A modifications influence immune infiltration in AS and guide subsequent treatments.

## 2. Materials and Methods

### 2.1. Data Collection

The transcriptome profiling datasets of 52 AS patients with active disease and 20 matched controls were obtained from publicly available datasets (http://www.ncbi.nlm.nih.gov/geo/) with the accession of GSE73754. The normalized matrix files for microarray data from the Illumina platforms were directly downloaded. We extracted a total of 21 m6A regulators from the dataset for corresponding analysis. These 21 m6A regulators are from a recently published paper [25], including eight Writers (*METTL3*, *ZC3H13*, *METTL14*, *RBM15B*, *CBLL1*, *WTAP*, *RBM15*, and *KIAA1429*), two Easers (*FTO* and *ALKBH5*), and 11 Readers (*YTHDC1*, *YTHDC2*, *ELAVL1*, *YTHDF1*, *LRPPRC*, *YTHDF2*, *FMR1*, *YTHDF3*, *HNRNPC*, *HNRNPA2B1*, and *IGF2BP1*).

### 2.2. Establishment of Random Forest Model and Support Vector Machine Model

Both random forest (RF) and support vector machine (SVM) are models for predicting the occurrence of AS. We evaluated the two models by using “Reverse Cumulative Distribution of Remainder”, “Boxplots of Remainder”, and the receiver operating characteristic (ROC) curve. Random forest as an integration and supervision model based on decision trees can be used for classification and regression. The RF model was established among the 21 m6A regulators by R statistical software with the package of “RandomForest” to predict the occurrence of AS. In our research, we first set the ntree and mtry values to 500 and 2, respectively. Then, we analyzed the point with the smallest cross-validation error in the RF model and selected the important disease-related m6A regulators. The SVM model can minimize a loss function to predict variables that are arranged between lower and upper estimated error bounds. The RF and SVM models were constructed by the R statistical software with the packages “RandomForest” and “KernLab”.

### 2.3. Nomogram Model of Significant m6A Regulators

We then used R to build a nomogram model to predict the risk of AS via significant candidate m6A regulators, paying attention to the calibration of the model. We also performed DCA and clinical impact curves to figure out whether the decisions based on the model were helpful to the patients. Moreover, ROC curves were built using the R package “pROC”.

### 2.4. AS Classification Based on Significant m6A Regulators

To explore the connection between the expression of 21 m6A regulators and AS subtypes, we applied unsupervised clustering with the R package “Consensus Cluster Plus” to discover distinct m6A modification patterns based on the expression of 21 m6A regulators; we raised the number of cluster *k* values from 2 to 9. The optimal number of clusters was estimated according to the consensus clustering algorithm, and the Pheatmap R package was used to build a heat map corresponding to consistent clustering and m6A expression.

### 2.5. Identification of Differentially Expressed Genes between Distinct m6A Subtypes and Classification of Subtypes Based on the DEGs

The “Limma” package in R was used to determine the Differentially Expressed Genes (DEGs) between different clusters in AS. A *p* value <0.05 was selected as the screening criterion. A consensus clustering method was used to classify AS into different genomic subtypes based on m6A-related DEGs.

### 2.6. Functional Enrichment Analysis of Differentially Expressed m6A-Related Genes

Along with the databases of the Gene Ontology (GO) and Kyoto Encyclopedia of Genes and Genomes (KEGG), the enrichment function of the m6A-related genes was analyzed and visualized by using the “Cluster Profiler” in R software. These analyses were performed based on these DEGs.

### 2.7. Generation of the m6A Gene Signature

To further explore the m6A patterns, we used principal component analysis (PCA) to calculate the m6A score for each sample. The process consists of two steps: the first step is to distinguish the m6A patterns; the second step is to calculate the m6A score according to the following formula [26, 27]: m6Ascore = ∑(PC1*i* + PC2*i*), where “*i*” represents DEG expression.

### 2.8. Evaluation of Immune Cell Infiltration

To evaluate the abundance of immune cells in AS, we used single-sample gene set enrichment analysis (ssGSEA) to calculate the scores of infiltrating immune cells and evaluate the correlation between the significant m6A regulators and the immune cells. The “GSVA” package was utilized to conduct the ssGSEA, and the “Pheatmap” package in R was used to plot the heat map between the infiltrating immune cells and the significant RNA N6-methyladenosine regulators.

### 2.9. Statistical Analysis

Pearson's chi-square test was used to analyze the correlations between Readers, Writers, and Erasers. “ConsensusClusterPlus” package in R was used to identify m6A subtypes and gene clusters. Kruskal-Wallis tests were adopted to compare the differences between clusters. All parametric analyses were based on two-tailed tests and *p* < 0.05 was set as the significance threshold. All data analyses were carried out using R software (version 4.1.2).

## 3. Results

### 3.1. The Landscape of the 21 m6A Regulators in AS

In the research, 21 m6A regulators were analyzed via the “Limma” package in R to find the differential expression levels between non-AS patients and AS patients. Eight significant m6A regulators (*WTAP*, *YTHDC1*, *CBLL1*, *HNRNPA2B1*, *METTL14*, *RBMX*, *ALKBH5*, and *IGFBP1*) were screened and visualized using a heat map and histogram. We found that *WTAP* and *YTHDC1* were over-expressed in AS patients, while the other significant m6A regulators displayed decreased expression in AS patients compared to non-AS patients (Figures 1(a) and 1(b)). The “RCircos” package in R was utilized to visualize the chromosomal positions of the 21 m6A regulators (Figure 1(c)). Spearman's correlation analysis of the 21 m6A RNA methylation modulators is shown in Figure 1(d).

### 3.2. Correlation between Writers, Readers, and Erasers in AS

To explore the gene expression levels among Writers, Readers, and Erasers, linear regression analyses were employed to analyze the correlation. *p* < 0.05 was set as the significance threshold and the correlation coefficient was set at 0.4. The expression levels of Writers and Readers, Erasers and Readers, and Writers and Readers could be found in (Figures 2(a)–2(l)). We found that the expression levels of *RBM15B*, *HNRNPA2B1*, *IGFBP1*, *RBMX*, and *YTHDC2* in AS patients had a significant positive correlation with *FTO*. Meanwhile, the expression levels of *LRPPRC*, *RBMX*, and *ELAVL1* displayed a positive correlation with *ALKBH5.* Furthermore, the results and analyses demonstrated positive correlations between Writers and Readers.

### 3.3. Establishment of Random Forest Model and Support Vector Machine Model

Eight candidate m6A regulators were chosen among a total of twenty m6A regulators. Then, we developed regression and support vector machine models to predict the occurrence of AS. Both the “Reverse Cumulative Distribution of residuals” and the “Boxplots of residuals” (Figures 3(a) and 3(b)) revealed that the RF model had minimal residuals. Following that, we further evaluated the model. The evaluation of receiver operating characteristic curve (ROC curve) (Figure 3(c)) and the AUC value of the ROC curve also indicated that the RF model was more appropriate than the SVM model (Figure 3(c)). Thus, we built a RF model based on the differentially expressed m6A-related genes between non-AS patients and AS patients (Figure 4(a)). We visualized these DEGs after classifying them according to their biological significance (Figure 4(b)). Eight candidate genes (*WTAP*, *YTHDC1*, *CBLL1*, *HNRNPA2B1*, *METTL14*, *RBMX*, *ALKBH5*, and *IGFBP1*) were selected based on the RF model with a score of greater than 2.

### 3.4. Establishment of the Nomogram Model

The “rms” in R package was used to establish a nomogram model based on the eight candidate m6A regulators for the purpose of forecasting the prevalence of AS patients (Figure 5(a)). It can be found from the calibration curves (Figure 5(b)) that the predictability of the nomogram model was accurate. The DCA curve showed that the red line (model line) remained above the gray line from 0 to 1, revealing that nomogram-based selections may benefit AS patients (Figure 5(c)). Furthermore, the clinical impact curve also indicated that the nomogram model had a significant predictive ability (Figure 5(d)). Additionally, ROC curve illustrated that our m6A regulators model got a better diagnostic power compared to other gene models (Figure 6).

### 3.5. Significant m6A Pattern Recognition Regulators for Two Distinct m6A Patterns

The consensus clustering method was used to identify distinct m6A patterns with eight significant candidate m6A regulators. We identified two m6A patterns using the R tool “Consensus Cluster Plus” (cluster A and cluster B) (Figures 7(a)–7(d)). The histogram and heat map were then generated to illustrate the differential expression of the eight distinct m6A regulators between the two clusters (Figure 7(e)). *YTHDC1*, *HNRNPA2B1*, and *IGFBP1* all had significantly higher expression levels in cluster A than those in cluster B. There were no significant differences in *WTAP*, *METTL14*, *CBLL1*, *RBMX*, or *ALKBH5* between cluster A and cluster B (Figure 7(f)). PCA clearly revealed that eight significant m6A regulators could distinguish the two m6A patterns (Figure 7(g)).

### 3.6. Classification of Subtypes Based on the DEGs and Evaluation of the m6A Gene Signature

In addition, we used the “Limma” package in R to analyze two m6A patterns. A total of 104 m6A-related DEGs were selected. To further explore the m6A patterns, AS patients were divided into different genomic subtypes based on the 104 m6A-related DEGs by using the “Consensus Cluster Plus”. Consistent with the m6A patterns, the gene patterns were also divided into two clusters (gene cluster A and gene cluster B) (Figures 8(a)–8(d)). A heat map is used in Figure 8(e) based on the expression of 104 DEGs in two gene patterns. Moreover, we tried to explore the expression differences of 21 m6A regulators between the two gene patterns, our research results revealed that *CBLL1*, *YTHDC1*, *HNRNPA2B1*, and *RBMX* had higher expression levels in gene cluster A, while *IGFNP1* had a higher expression level in gene cluster B (Figure 8(f)). To quantify the m6A patterns, PCA algorithms were utilized to calculate the m6A score for each sample. Subsequently, we compared the m6A score between the two distinct m6A gene clusters and the m6A clusters. It can be seen from the results that the m6A score in cluster A or gene cluster A was higher than that in cluster B or gene cluster B (Figures 8(g) and 8(h)).

### 3.7. Analyses of Immune Characterization and Functional Enrichment

We performed the GO and KEGG analyses to understand the possible mechanism of these DEGs in AS. GO analysis suggested that DEGs mainly concentrated in the processes of heme metabolic, porphyrin containing compound metabolic, tetrapyrrole metabolic, hydrogen peroxide metabolic, hydrogen peroxide catabolic, the modification of mitochondrial matrix, mitochondrial inner membrane and hemoglobin complex, the activity of ubiquitin-protein transferase, ubiquitin-protein ligase, and oxidoreductase (Figure 9(a)). Moreover, KEGG analysis demonstrated that DEGs mainly concentrated in porphyr in metabolism, longevity regulating pathway, glycine, serine and threonine metabolism, mTOR signaling pathway, as well as p53 signaling pathway (Figure 9(b)). In addition, ssGSEA was applied to calculate the abundance of immune cells in AS and to evaluate the correlation between the eight distinct m6A regulators and immune cells. The result of the heat map displayed the correlation between the eight distinct m6A regulators and immune cells (Figure 10(a)). We could conclude that *HNRNPA2B1* had positive correlations with numerous immune cells. Then, the two groups (high *HNRNPA2B1* expression and low HNRNPA2B1 expression) were used to evaluate the differential immune cell infiltration (Figure 10(b)). The results indicated that patients with high *HNRNPA2B1* expression had increased immune cell infiltration compared to those with low *HNRNPA2B1* expression. Furthermore, we tried to evaluate the correlation between m6A clusters and differential immune cell infiltration (Figure 10(c)). The results showed that the two significant m6A patterns were consistent with activated CD4 T cell immunity, activated CD8 T cell immunity, and MDSC immunity. Cluster A was linked to activated CD4 T cell immunity and activated CD8 T cell immunity, while cluster B had a correlation with the immunity of MDSC that has been linked to immunosuppressive functions, which indicated that cluster A might be related to AS. In addition, we explored the relationship between gene clusters and differential immune cell infiltration, and the result was consistent with the correlation between m6A cluster A and differential immune cell infiltration (Figure 11(a)). The Sankey diagram shows the changes in m6A cluster, gene cluster, and m6A score (Figure 11(b)).

### 3.8. Role of m6A Patterns in Distinguishing AS

We explored the correlation between m6A patterns and risk genes in order to obtain a better understanding of the association between m6A patterns and AS (Figures 11(c) and 11(d)). We noticed that the expression levels of *CD3D*, *PTGER4*, and *BACH2* were significantly higher in cluster A or gene cluster A than those in cluster B or gene cluster B, indicating that cluster A or gene cluster A may be strongly associated with AS.

## 4. Discussion

AS is a complex and potentially debilitating disease with an insidious onset, which would progress to radiation sacroiliitis in several years. According to the research papers published in recent years, m6A regulators reportedly play an important role in biological processes. However, the role of m6A regulators in AS remains unknown.

Through differential expression analyses, we identified eight significant m6A regulators among 21 m6A regulators in AS patients and non-AS patients. Eight candidate m6A regulators (*WTAP*, *YTHDC1*, *CBLL1*, *HNRNPA2B1*, *METTL14*, *RBMX*, *ALKBH5*, and *IGFBP1*) were extracted from the RF model to predict the occurrence of AS. Following that, we made a nomogram based on the eight candidate m6A regulators, and we used the DCA curve to see how the nomogram model benefited the AS patients.

m6A is a methylated modification generated by methylating the sixth position N of adenine on messenger RNA (mRNA) using a methyltransferase complex (*MTC*) [28, 29]. *WTAP* is a nuclear protein that functions as the partner of Wilms' tumor 1 (WT1) [30]. *WTAP* deletion has been verified to be embryonically fatal [31], indicating its critical biological role in vertebrate development. Meanwhile, as an important part of the MTC, WTAP can promote the formation of m6A [32]. Within the cytoplasm, YTHDF1 promotes the initiation of translation and the decay of m6A-dependent mRNA. Within the nucleus, it binds to m6A-modified RNAs and facilitates splice site selection [33]. *CBLL1* is an evolutionarily conserved E3 ubiquitin ligase containing a RING-finger domain, and extensive studies have demonstrated that *CBLL1* plays an important role in tumorigenesis [34]. *HNRNPA2B1* regulates Wnt signaling transcriptional activity by regulating the stability of *TCF7L2* mRNA, and it is related to tumor growth [24, 35]. Mass spectrometry has shown that *METTL14* works to make m6A methylation, and it can form a stable heterodimer. *METTL14* is a key RNA-binding scaffold that plays a crucial role in recognition of substrate RNAs [36]. *RBMX* was initially identified as a component of the spliceosome and is involved in alternative splicing. RBMX has been rediscovered in recent years to participate in DNA damage repair, sister chromatid cohesion, and the assembly of higher-order ribonucleoprotein complexes [37–40]. Human AlkB homolog H5 (*ALKBH5*) could demethylate long noncoding RNAs, promote cancer cell self-renewal, or regulate autophagy in malignancies, playing a fundamental role in noncancerous reproductive system illnesses in humans [41]. Insulin-like growth factor binding protein-1 (*IGFBP-1*) is a member of the insulin-like growth factor (IGF) system. *IGFBP-1*'s biological effects in cancer have been discovered to be reliant on its phosphorylation status, as well as on IGF-dependent and -independent pathways [42]. Increasing studies have proved that the eight m6A regulators have a correlation with the occurrence of cancer. However, no reports are available on the relationship between the eight candidates m6A regulators and AS. We hope that the selected eight distinct m6A regulators can provide a direction for future clinical research.

Furthermore, two clusters were divided based on the eight distinct m6A regulators. Compared with cluster B, *ALKBH5* and *FTO* showed higher expression levels in cluster A in our study. Then PCA was established to distinguish the m6A patterns. Additionally, 104 DEGs were obtained based on the two m6A clusters, GO terms, and KEGG pathway analysis. This study revealed that 104 m6A-related DEGs mainly concentrated in the processes of heme metabolic, porphyrin containing compound metabolic, tetrapyrrole metabolic, hydrogen peroxide metabolic, hydrogen peroxide catabolic, the modification of mitochondrial matrix, mitochondrial inner membrane and hemoglobin complex, the activity of ubiquitin-protein transferase, ubiquitin-protein ligase, and oxidoreductase. Moreover, KEGG analysis demonstrated that DEGs mainly concentrated in porphyrin metabolism, longevity regulating pathway, glycine, serine and threonine metabolism, mTOR signaling pathway, as well as p53 signaling pathway. Besides, we further divided the AS patients into two genomic subtypes (gene cluster A and gene cluster B) based on the 104 DEGs. Then, the m6A score for each sample was calculated by using PCA algorithms, and comparisons were made between the significant m6A gene clusters and m6A clusters. The results showed that the m6A score in cluster A or gene cluster A was higher than that in cluster B or gene cluster B.

AS is a chronic inflammatory disease of unknown etiology in which the innate immune system plays a dominant role and is characterized by abnormal activation of innate immune cells. When considering the ssGSEA analysis, we also discovered that the two significant m6A patterns were consistent with activated CD4 T cell immunity, activated CD8 T cell immunity, and MDSC immunity. The immunity of MDSC, on the other hand, has been linked to immunosuppressive functions [43]. In the previous studies, several risk genes (*TYK2*, *BACH2*, *IL6R*, *IL7R*, *IL12B*, *IL27*, *NKX2*, and *PTGER4*) play a vital role in the development of AS. Cluster A was found to be more associated with activated CD4 T cell immunity, activated CD8 T cell immunity, and lower MDSC immune infiltration, compared with cluster B, which implied that cluster A may be related to AS.

In short, we used the consensus clustering method to discover two m6A patterns (cluster A and cluster B) based on the eight significant m6A regulators and to identify two gene patterns (gene cluster A and gene cluster B) based on the 104 DEGs. Cluster A and gene cluster A were found to be enriched in activated CD4 T cell immunity, activated CD8 T cell immunity, and MDSC immunity by ssGSEA, implying that cluster A and gene cluster A may be associated with AS. Then m6Ascore was calculated based on the m6A modification, and the Sankey diagram was used to attribute changes among m6A clusters, m6A gene clusters, and m6A score.

Currently, there are few articles on the relationship between m6A regulators and AS, therefore, our findings have provided novel ideas for identifying different AS phenotypes and promoting personalized diagnosis in the future. The aim of our study is to find out more about the role of m6A regulators in AS. However, there are still some limitations in our study. For instance, our model is not validated in an independent data set due to a lack of datasets with m6A regulators in the public database. Another problem is that our clinical data is relatively incomplete. Moreover, the sample data we utilized for our study are obtained retrospectively, so all analyses are conducted on public databases. Inevitably, the research outcomes might have been partial as a result of the inherent case selection bias. To confirm our results, larger prospective studies as well as in vitro and vivo experiments are needed.

## 5. Conclusion

To conclude, we build in our research a nomogram model that accurately predicts the occurrence of AS by using eight distinct m6A regulators. Additionally, we find two significant m6A patterns and two gene clusters based on eight important m6A regulators and DEGs, and our research findings show that cluster A and gene cluster A may be associated with AS. Our work offers a foundation for further research on various AS phenotypes, providing more insight into the future diagnosis and treatment of AS.

## Figures and Tables

**Figure 1:** Landscape of the 21 RNA N6-methyladenosine (m6A) regulators in AS. (a) Differential expression histogram of the 21 m6A regulators identified between non-AS and AS patients. (b) Expression heat map of the 21 m6A regulators between non-AS and AS patients. (c) Chromosomal positions of the 21 m6A regulators. (d) Spearman's correlation analysis of the 21 m6A RNA methylation modulators in AS patients ^∗^*p* < 0.05, ^∗∗^*p* < 0.01, and ^∗∗∗^*p* < 0.001.

**Figure 2:** Correlation between Writers, Readers, and Erasers in AS patients (a–l). Writer genes: *WAP1*, *RBM15*, *RBM15B*, *METTL14*, *METTL3*, *KIAA1429*, *CBLL1*, and *ZC3H1*; Eraser genes: *ALKBH5* and *FTO*; Reader genes: *YTHDC1*, *YTHDC2*, *ELAVL1*, *YTHDF1*, *LRPPRC*, *YTHDF2*, *FMR1*, *YTHDF3*, *HNRNPC*, *HNRNPA2B1*, and *IGF2BP1*.

**Figure 3:** Establishment of random forest model and support vector machine model. (a) The RF and support vector machine (SVM) residual distributions are plotted using the reverse cumulative distribution of residuals. (b) The residual distribution of the RF and SVM models is depicted using boxplots. (c) ROC curves demonstrate the accuracy of the RF model and the SVM model.

**Figure 4:** Random Forest (RF) Model construction. (a) The RF model is established among the 21 m6A regulators. (b) The importance of the eight RNA N6-methyladenosine regulators based on the RF model.

**Figure 5:** Establishment of the nomogram model. (a) Construction of the nomogram model based on the five candidate RNA N6-methyladenosine regulators. (b) Predictive ability of the nomogram model as revealed by the calibration curve. (c) Decisions based on the nomogram model may benefit AS patients. (d) Clinical impact of the nomogram model as assessed by the clinical impact curve.

**Figure 6:** Validation of nomogram model in the diagnostic value. (a) ROC curve analysis of nomogram model. (b) ROC curve analysis of gene PUM1 model. (c) ROC curve analysis of gene ZFP91 model.

**Figure 7:** Consensus clustering of the 8 distinct RNA N6-methyladenosine (m6A) regulators in AS patients. (a) The consensus clustering matrix at *k* = 2. (b) The consensus clustering matrix at *k* = 3. (c) CDF curve for *k* = 2 to 9. (d) The relative variation of the area under the CDF curve that *k* is from 2 to 9. (e) Expression heat map of the 8 significant m6A regulators in cluster A and cluster B. (f) Differential expression histogram of the 8 significant m6A regulators in cluster A and cluster B. (g) Principal component analysis on the expression profiles of the 8 significant m6A regulators that shows a remarkable difference in transcriptomes between the two m6A patterns ^∗^*p* < 0.05, ^∗∗^*p* < 0.01, and ^∗∗∗^*p* < 0.001.

**Figure 8:** Consensus clustering of the 104 RNA N6-methyladenosine (m6A)-related DEGs in AS patients. (a) The consensus clustering matrix at *k* = 2. (b) The consensus clustering matrix at *k* = 3. (c) CDF curve for *k* = 2 to 9. (d) The relative variation of the area under the CDF curve that *k* is from 2 to 9. (e) Expression heat map of the 104 m6A-related DEGs in gene cluster A and gene cluster B. (f) Differential expression histogram of the 8 significant m6A regulators in gene cluster A and gene cluster B. (g) Differences in m6A score between cluster A and cluster B. (h) Differences in m6A score between gene cluster A and gene cluster B. ^∗^*p* < 0.05, ^∗∗^*p* < 0.01, and ^∗∗∗^*p* < 0.001.

**Figure 9:** GO and KEGG analyses of 104 DEGs. (a) Barplot displayed the potential mechanism underlying the effect of the 104 m6A-related Differentially Expressed Genes (DEGs) on the occurrence and development of AS. (b) The significant KEGG pathways of these m6A-related genes and DEGs.

**Figure 10:** Single sample gene set enrichment analysis. (a) Correlation between infiltrating immune cells and the 8 significant RNA N6-methyladenosine regulators. (b) Differences in the abundance of infiltrating immune cells between high and low *HNRNPA2B1* expression groups. (c) Differential immune cell infiltration between m6A cluster A and m6A cluster B. ^∗^*p* < 0.05, ^∗∗^*p* < 0.01, and ^∗∗∗^*p* < 0.001.

**Figure 11:** Role of RNA N6-methyladenosine (m6A) patterns in distinguishing AS. (a) Differential immune cell infiltration between gene cluster A and gene cluster B. (b) Sankey diagram showing the relationship between m6A patterns, m6A gene patterns, and m6A scores. (c) Differential expression levels of *TYK2*, *PTGER4*, *CD3D*, *IL23R*, *KIF21B*, *ERAP1*, *ERAP2*, *BACH2*, and *CXCR2* between cluster A and cluster B. (d) Differential expression levels of *TYK2*, *PTGER4*, *CD3D*, *IL23R*, *KIF21B*, *ERAP1*, *ERAP2*, *BACH2*, and *CXCR2* between gene cluster A and gene cluster B. ^∗^*p* < 0.05, ^∗∗^*p* < 0.01, and ^∗∗∗^*p* < 0.001.

## Data Availability

Data generated or used in this study are available from the corresponding author upon reasonable request.

## Abbreviations

AS: Ankylosing spondylitis
GEO: Gene Expression Omnibus
HLA: Human Leukocyte Antigen
ROC: Receiver operating characteristic curve
AUC: Area under control
GO: Gene ontology
KEGG: Kyoto encyclopedia of genes and genomes
PCA: Principal components analysis
DCA: Decision curve analysis
RF: Random forest
SVM: Support vector machine
SPA: Spondyloarthropathies
DEG: Differentially expressed genes
ssGSEA: Single sample gene set enrichment analysis
m6A: N6-methyladenosine
